The article "Analysis of the Mechanism and Safety of Bisphosphonates in Patients with Lung Cancer and Bone Metastases" was retracted in 2023. Reason: concerns about the peer review.

# Analysis of the Mechanism and Safety of Bisphosphonates in Patients with Lung Cancer and Bone Metastases

**DOI:** 10.1155/2021/5343104

**Published:** 2021-12-13

**Authors:** Gao Zhang, Hu Gong, Hanqiao Xu

**Affiliations:** ^1^Department of Oncology, General Hospital of Central Theater Command of Chinese People's Liberation Army, Hubei Wuhan 430070, China; ^2^Department of Orthopedics, Wuhan Sixth Hospital, Affiliated Hospital of Jianghan University, Hubei Wuhan 430015, China; ^3^Department of Thoracic Surgery, Wuhan Sixth Hospital, Affiliated Hospital of Jianghan University, Hubei Wuhan 430015, China

## Abstract

**Objective:**

To explore the mechanism and safety of bisphosphonates in patients with lung cancer and bone metastases.

**Method:**

A total of 104 patients with lung cancer and bone metastases in our hospital were selected and randomly divided into two groups: control group (*n* = 54) and research group (*n* = 50). Chemotherapy was given to the control group, and the research group was treated with bisphosphonate drugs. The quality of life, HAMA, HAMD score, VAS score, treatment effect, serum calcium and KPS score, inflammatory factor levels, and immune function were compared between the two groups.

**Result:**

The quality of life in both groups was significantly increased (*P* < 0.05). The HAMA and HAMD scores of the research group decreased significantly than those of the control group after treatment (*P* < 0.05). The VAS scores of the two groups were significantly reduced (*P* < 0.05). The effective rates of treatment in the control group and the research group were 81.5% and 96.0%, respectively. Serum calcium was significantly decreased, and KPS score was significantly increased at weeks 1 and 6 after treatment, and the change was more obvious in the research group (*P* < 0.05). The levels of inflammatory factors in the two groups were significantly reduced, and the immune indicators were significantly increased.

**Conclusion:**

Bisphosphonates have good effect on patients with lung cancer and bone metastases, which can improve anxiety and depression, reduce pain score, improve serum calcium level and immune function, and reduce inflammatory response. Therefore, bisphosphonate drug therapy is worth widely used.

## 1. Preface

The clinical incidence of lung cancer is relatively high and the common metastatic site is bone. Patients with bone metastases have obvious symptoms of pathological fractures, spinal cord compression, bone pain, and hypercalcemia. It has a significant influence on patients' quality of life, and it will put patients' lives in jeopardy as the condition advances [1]. At the moment, clinical treatment consists mostly of bisphosphonates, radiation, and surgery. Bisphosphonate medicines decrease bone breakdown and resorption, while also lowering blood calcium levels, which aids in the healing of osteolytic lesions to a certain degree [2]. Third-generation and second-generation bisphosphonate medications are the most widely used clinically, with zoledronate sodium and ibandronate sodium representing third-generation bisphosphonates, respectively, and pamidronate sodium representing second-generation bisphosphonates. In comparison to the second generation of bisphosphonates, the third generation of bisphosphonates has a superior therapeutic impact; however, there are few clinical findings on this point [3, 4].

104 patients admitted to our hospital were chosen for this research to investigate the therapeutic mechanism and safety of bisphosphonates in order to alleviate clinical symptoms, reduce discomfort, and enhance prognosis. The relevant contents are reported as follows.

## 2. Information and Method

### 2.1. General Information

104 patients in our hospital were randomly divided into two groups. There are 54 patients in the control group, age 20-72 years, mean age 68.2 ± 2.9 years, 28 female, 26 male, disease duration 1-5 years, mean disease duration 3.1 ± 0.6 years, 54 patients, stage IV 18, and stage III 36. There are 50 patients in the research group, age 20-71 years, mean age 68.1 ± 2.8 years, 24 females and 26 males, duration of disease 1-5 years, mean duration of disease 3.2 ± 0.7 years, 50 patients, stage IV 16, and stage III 34. Inclusion criteria [5] are as follows: (1) no participation in other clinical studies during the study period; (2) age is older than 18 years; (3) patient was diagnosed, (4) meeting the diagnostic criteria; (5) stable vital signs and acceptable for prognostic follow-up; and (6) expected survival cycle more than 12 months. Exclusion criteria are as follows: (1) patients with other cancerous lesions; (2) autoimmune system diseases; (3) hepatic, renal, or coagulation dysfunction; (4) patients with psychiatric abnormalities; and (5) patients with incomplete clinical information and low adherence. The study subjects agreed to the study, the data were comparable (*P* > 0.05), and the hospital ethics committee agrees it.

### 2.2. Method

The control group underwent chemotherapy and was administered gemcitabine at a dose of 1000 mg/m^2^. On the first and eighth days, add 25 mg/m^2^ cisplatin. Each cycle lasts three weeks, and six cycles of continuous therapy are performed.

The research group received zoledronic acid (GuoPharm quantification H20041955, manufacturer: GuoPharm Group Guorui Pharmaceutical Co., Ltd.) in 100 ml of saline for a total of 15-minute intravenous drip, one time per week for three weeks, followed by bone imaging and X-ray review following two cycles of continuous treatment.

### 2.3. Observation Indicators

*Quality of survival* [6]: the FACT-G-V score was applied to evaluate the quality of survival, containing indicators of functional status, physical status, emotional status, and family/social status.

*HAMA and HAMD scores* [7]: use Hamilton Anxiety Scale (HAMA) and Depression Scale (HAMD) to evaluate the degree of anxiety and depression. There are a total of 15 items. Score 10 means the improvement in anxiety and depression is most obvious.

*VAS score* [8]: apply pain scale (VAS) to evaluate the degree of pain in patients. The total score is 10 points. Score 1 means the pain is most lower.

*Treatment effect* [9]: ineffective: new lesions developed or existing lesions became larger after therapy; effective: after treatment, calcification developed or lesions greatly decreased in size. After therapy, lesions become calcified or all metastases disappear. The effective rate is calculated as the total of all instances that are both remarkably effective and effective. Multiply by the total number of instances and divide by 100%. A greater effective rate indicates a more pronounced therapeutic impact. For the KPS score and serum calcium [10], 3 ml fasting venous blood was extracted, centrifuged at 3500 rpm for 10 minutes, serum collected, and the calcium level determined using the selective electrode technique. The necessary procedures were carried out in accordance with the instructions. The greater the therapeutic impact, the closer the results converged to normal levels. For the inflammatory factor levels [11], 3 ml fasting venous blood was drawn and centrifuged at 3500 rpm for 10 minutes to obtain serum. Enzyme-linked immunoassay was used to detect the levels of interleukin-6 (IL-6), C-reactive protein (CRP), and tumor necrosis factor-*α* (TNF-*α*).

*Immune function* [12, 13]: flow cytometry was applied to antibody labeling, CD4+ and CD8+ levels were detected, and CD4+/CD8+ was calculated.

### 2.4. Statistical Method

Statistical analysis was performed with SPSS19.0. The statistical data adopts two-sided test, and *P* < 0.05 indicates that the difference is statistically significant. Quantitative data is expressed by (*x* ± *s*) and compared by *t*-test. ANOVA was used to compare samples from three different groups. LSD compared all of the findings two by two. The *X*^2^ test was used to assess qualitative data. GraphPad Prism was used to create the graphs.

## 3. Result

### 3.1. Survival Quality

The survival quality increased after treatment, and survival quality of the research group increased more significantly both in functional status, physiological condition, emotional state, and emotional state (*P* < 0.05) (Table 1).

### 3.2. Comparison of Scores of HAMA and HAMD

After treatment, HAMA and HAMD scores in both groups decreased significantly, and the differences between two groups were statistically significant (*P* < 0.05) (Table 2).

### 3.3. Comparison of VAS Scores

After treatment, VAS scores of the two groups decreased significantly, and the difference was statistically significant (*P* < 0.05) (Table 3).

### 3.4. Comparison of Treatment Effect

The effective rate of two groups was 81.5% and 96.0%, respectively. The effective rate of the research group was higher than that of control group, and the difference was significant (*P* < 0.05) (Figure 1).

### 3.5. KPS Scores and Serum Calcium Levels Are Compared

At 1 week and 6 weeks following therapy, serum calcium levels dropped dramatically, while KPS scores rose significantly in both groups. When compared to the control group, the alterations in the research group were more apparent, and there was a significant difference (*P* 0.05). (Figure 2).

### 3.6. Comparison of Inflammatory Factor Level

The levels of inflammatory factors were significantly reduced. However, the decrease in the research group was more obvious (*P* < 0.05) (Figure 3).

### 3.7. Comparison of Immune Function

The immune indexes were significantly higher in both groups after treatment. However, the increase of the research group was more obvious, and the difference was statistically significant (*P* < 0.05) (Figure 4).

## 4. Discussion

It is clinically proven that lung cancer bone metastasis is the main site of bone, and bone metastases by themselves are not life-threatening in the short term. They may increase the risk of adverse outcomes, such as hypercalcemia and pathological fractures, if left untreated [14–16]. The most common clinical symptom is osteolytic damage. The use of radiation and pain medication in the clinic will raise the likelihood of side effects and a poor prognosis, as well as the occurrence of bone metastases, which will restrict treatment options [17, 18]. Bisphosphonates are increasingly being employed in the therapeutic treatment of individuals with bone metastases from malignant malignancies. There are also clinical trials underway to demonstrate the drug's therapeutic efficacy, which will include a considerable antitumor effect on the quantity and activity of osteoclasts, as well as an effective suppression of tumor bone metastasis [19, 20]. At present, in the level of medical progress and development, many scholars put more effort on the therapeutic effect of the third-generation bisphosphonate drug, and the study confirmed that the third-generation bisphosphonate drug 90.8% disease remission rate is higher compared with the second-generation bisphosphonate drug 83.9% disease remission rate [21]. However, there are few clinical studies on bisphosphonates for the treatment of a particular disease, mainly for prostate cancer and breast cancer [22]. Bisphosphonates will inhibit bone and tumor cell binding, stop malignant tumor progression, and play an important role in reducing pain [23].

Tumor cells will degrade the bad bone apoptotic component, osteoclasts will be activated, osteolysis will be seen, and bone metastases will damage bone, resulting in an increase in blood calcium levels [24]. The study evaluated the therapeutic effectiveness of bisphosphonate medicines in eligible individuals with lung cancer and bone metastases. The study's results indicated that treatment efficacy rates were 81.5 percent and 96.0 percent in the control and research groups, respectively. Serum calcium levels decreased considerably after 1 and 6 weeks of treatment, but the KPS score increased significantly. The data indicate that, when compared to the radiation index, bisphosphonate medications are more successful and beneficial for improving patients' blood calcium levels, implying that they may be used as a safe and effective treatment technique for clinical symptoms. The primary symptom is bone discomfort. Certain patients will experience worry, despair, and other bad feelings as a result of the pain being aggravated. Patients' pain complaints improved dramatically after bisphosphonate medication, which may enhance patients' adherence to treatment [25].

At present, atmospheric pollution is becoming more and more serious, the incidence of lung cancer is increasing, and some patients do not understand the causes of the disease and the principles of treatment, and they worry about the prognosis, which can lead to negative emotions. Patients' symptoms were greatly improved after therapy, which aided in the eradication of negative feelings in the patients [26]. Both groups' quality of life improved dramatically following therapy, according to the findings. HAMA and HAMD scores were considerably lower in both groups, with the research group's scores being significantly lower (*P* 0.05). The findings reveal that, as compared to radiation indices, bisphosphonate medication treatment may significantly enhance patients' negative feelings, as well as their overall survival functions. In addition, the results showed that bisphosphonates played an important role in improving immune function and reducing inflammatory factors. The feasibility and value of clinical application are high.

In conclusion, bisphosphonate medication for lung cancer bone metastases has an optimum impact, improving anxiety and sadness while reducing pain ratings, improving serum calcium levels and immunological function, and reducing inflammatory reactions. Therefore, bisphosphonate drug therapy is worthy of wide application.

## Figures and Tables

**Figure 1:** Comparison of the treatment effect.

**Figure 2:** Comparison of serum calcium and KPS scores.

**Figure 3:** Comparison of inflammatory factor levels.

**Figure 4:** Comparison of immune function.

**Table 1:** Comparison of quality of survival.

Groups	Number of cases	Functional status		Physiological condition		Emotional state		Family/social situation	
		Before	After t	Before	After	Before	After	Before	After
Control subjects	54	19.1 ± 5.2	15.1 ± 4.4	21.4 ± 8.2	17.2 ± 6.0	18.4 ± 4.6	15.6 ± 5.3	20.2 ± 7.7	16.0 ± 5.2
Research group	50	19.2 ± 5.1	13.2 ± 4.0	21.2 ± 8.0	14.2 ± 0.8	18.2 ± 4.5	13.2 ± 4.6	20.3 ± 7.5	14.2 ± 5.0
*T*	/	0.524	16.854	1.754	18.524	0.874	16.382	0.854	17.985
*P*	/	>0.05	<0.05	>0.05	<0.05	>0.05	<0.05	>0.05	<0.05

**Table 2:** Comparison of HAMA and HAMD scores.

Groups	Case number	HAMA (points)		HAMD (points)	
		Before treatment	After treatment	Before treatment	After treatment
Control subjects	54	23.2 ± 3.4	17.3 ± 5.1	22.6 ± 3.6	18.7 ± 3.4
Research group	50	23.1 ± 3.5	13.6 ± 5.3	22.4 ± 3.8	14.1 ± 3.2
*T*	/	0.524	16.854	1.985	15.742
*P*	/	>0.05	<0.05	>0.05	<0.05

**Table 3:** Comparison of VAS scores.

Groups	Number of cases	VAS score (points)	
		Before treatment	After treatment
Control subjects	54	7.4 ± 1.9	5.2 ± 1.6
Research group	50	7.3 ± 2.0	4.3 ± 1.2
*T*	/	0.896	17.582
*P*	/	>0.05	<0.05

## Data Availability

The data used to support the findings of this study are included within the article.
